The article "Robust LQR-Based Neural-Fuzzy Tracking Control for a Lower Limb Exoskeleton System with Parametric Uncertainties and External Disturbances" was retracted in 2023. Reasons: signs of a paper mill; compromised peer review; unreliable results or conclusions.

# Robust LQR-Based Neural-Fuzzy Tracking Control for a Lower Limb Exoskeleton System with Parametric Uncertainties and External Disturbances

**DOI:** 10.1155/2021/5573041

**Published:** 2021-06-11

**Authors:** Jyotindra Narayan, Santosha K. Dwivedy

**Affiliations:** Department of Mechanical Engineering, Indian Institute of Technology Guwahati, Guwahati 781039, India

## Abstract

The design of an accurate control scheme for a lower limb exoskeleton system has few challenges due to the uncertain dynamics and the unintended subject's reflexes during gait rehabilitation. In this work, a robust linear quadratic regulator- (LQR-) based neural-fuzzy (NF) control scheme is proposed to address the effect of payload uncertainties and external disturbances during passive-assist gait training. Initially, the Euler-Lagrange principle-based nonlinear dynamic relations are established for the coupled system. The input-output feedback linearization approach is used to transform the nonlinear relations into a linearized state-space form. The architecture of the adaptive neuro-fuzzy inference system (ANFIS) and used membership function are briefly explained. While varying mass parameters up to 20%, three robust neural-fuzzy datasets are formulated offline with the joint error vector and LQR control input. Thereafter, to deal with external interferences, an error dynamics with a disturbance estimator is presented using an online adaptation of the firing strength matrix. The Lyapunov theory is carried out to ensure the asymptotic stability of the coupled human-exoskeleton system in view of the proposed controller. The gait tracking results for the proposed control scheme (RLQR-NF) are presented and compared with the exponential reaching law-based sliding mode (ERL-SM) controller. Furthermore, to investigate the robustness of the proposed control over LQR control, a comparative performance analysis is presented for two cases of parametric uncertainties and external disturbances. The first case considers the 20% raise in mass values with a trigonometric form of disturbances, and the second case includes the effect of the 30% increment in mass values with a random form of disturbances. The simulation runs have shown the promising gait tracking aspects of the designed controller for passive-assist gait training.

## 1. Introduction

Over the last two decades, an increasing number of neurological disorders such as stroke, spinal cord injury, and Parkinson's disease have been observed in different age groups. The World Health Organization (WHO) reported “stroke” as one of the principal reasons for nearly 5 million people's fatality through 2000-2016 and the third pioneering source of debility throughout the world [1]. To address the concerns of motor functionality in the lower body caused by neurological disorders, researchers have developed many robot-based lower limb exoskeleton devices to produce therapeutic effects during walking [2, 3]. In a recent work by Kalita et al. [4], a systematic yet comprehensive review has been carried out on the state-of-the-art developments of such multijoint and single-joint exoskeleton devices for gait rehabilitation, mobility aid, and strength amplification.

A well-known treadmill-oriented exoskeleton, LOPES [5], has been developed with a 2D translatable pelvis segment, two active hip joints, and an active knee joint for lower limb rehabilitation. The system was controlled to supervise or follow the subjects using “robot-in-charge” and “subject-in-charge” modes. Bortole et al. [6] designed a 6-DOF lower limb exoskeleton for overground training of stroke subjects with a body height of 1.50-1.95 m and a body mass of 100 kg. Hsieh et al. [7] proposed a soft exoskeleton design for preswing gait training of subjects with weak muscles, where a single actuator with a pulley-slider arrangement is used to drive the lower limb joints. The prototype is developed and clinically investigated with seven subjects. In a study on a parallel mechanism-based lower limb rehabilitation, Rastegarpanah et al. [8] investigated the performance of a 6-DOF robot by executing foot trajectories of 20 healthy subjects. Furthermore, the same prototype was tested for eight poststroke patients while carrying out three exercises, i.e., hip flexion/extension, ankle dorsiflexion/plantarflexion, and marching [9]. Aggogeri et al. [10] presented a modular and reconfigurable mechanism for rehabilitating ankle joints of different subjects. Cestari et al. [11] introduced the ATLAS exoskeleton to assist the children during flexion/extension of the hip, knee, and ankle joints. At the preliminary level, a dummy with body features of a 10-year-old child was used to test the exoskeleton system. Patané et al. [12] proposed a multijoint exoskeleton, WAKE-up, to rehabilitate the knee, ankle, and foot of the pediatric subjects with neurological disorders. The device was tested with four healthy children and three children with cerebral palsy. To amplify human endurance while carrying heavy loads, BLEEX [13] (7-DOF/limb) was developed with intelligent and adaptable robot-based strategies where linear hydraulic actuators were used for the actuation of 4-DOF. Recently, Ji et al. [14] introduced a wearable exoskeleton, SIAT-WEXv2, to support the user's waist and bones while lifting heavy objects in construction and logistic industries by providing an assistive output of 28 N.

To augment the rehabilitation devices' performance, the appropriate control schemes are designed by the researchers for executing repetitive gait movements. The control architecture required for the exoskeleton systems poses extra complexity over the conventional robotic arm control due to the sophisticated mechanical configuration, complex motion trajectory, and human involvement. The researchers, in the literature, have regarded the predefined gait tracking control as the basis of every control scheme for exoskeleton systems, where the joint movements of the lower limb could be estimated using gait analysis experiments [15, 16, 17]. Although the exoskeleton systems exploit the gait of healthy humans to replicate the same using predefined trajectory control schemes, however, in practice, they are unable to attain the proper gait trajectory because of the parametric uncertainties and external disturbances (PUEDs). Therefore, various robust control strategies have been designed to deal with the limitations of classical trajectory tracking control in lower limb exoskeleton systems [18, 19, 20, 21, 22, 23]. Ajayi et al. [18] proposed a bounded control scheme for the rehabilitation of the knee ankle joint of a user in a sitting position. The stability of the control law and convergence analysis of the gain observer is validated with the Lyapunov theory. The simulation results are presented without and with the effect of the human interaction torque. Yang et al. [19] presented a sliding mode control (SMC) scheme where a second-order command filter-aided backstepping is incorporated to avert the “explosion of complexity.” Moreover, the fuzzy logic is exploited to counter the chattering issues of the control scheme during the estimation of structured and unstructured uncertainties. In another work on robust control, Long et al. [20] presented a hybrid strategy where SMC is augmented with a cerebellar model articulation controller (CMAC) to predict the motion intent of the subject. The optimized sliding surface of the SMC is estimated using the genetic algorithm to improve the effectiveness of the proposed control scheme. Liu et al. [21] introduced an event-triggered SMC for effective tracking of the reference trajectory using a lower limb exoskeleton system with PUEDs. In another work to address the model uncertainties and the unintended subject's response, Wu et al. [22] proposed an adaptive control scheme for a 3-DOF lower extremity rehabilitation device. Working on the decoupled control strategy, Sun et al. [23] designed a reduced-order adaptive fuzzy approach and implemented it on a two-link exoskeleton system for lower limb rehabilitation.

Furthermore, in recent times, robust intelligent control schemes have gain popularity to address the adverse effects of PUEDs with effective approximation features. A neural network (NN) along with a time-delay evaluation-based control scheme is proposed by Zhang et al. [24] to realize the desired gait trajectory for a simulated model of a 10-DOF exoskeleton. The performance of the designed control scheme is investigated by comparing the classical PD control scheme. Narayan and Dwivedy [25] proposed a neuro-fuzzy compensator for PID control to deal with the system's known and unknown uncertainties during passive gait rehabilitation of a human child. The controller is found to be more robust towards external disturbances over payload uncertainties. Chen et al. [26] proposed a disturbance estimator-based subject-cooperative control for a weight-reinforced active-assist rehabilitation device. They computed the interaction torques using a backpropagation neural network-aided disturbance observer and proved the stability using the Lyapunov theory. In a recent work by Han et al. [27], time-delay estimator-aided computed torque control is designed to deal with PUEDs of a lower limb exoskeleton system. Moreover, an adaptive radial basis function neural network (RBFNN) is utilized to compensate for the time-delay error.

On the other hand, few researchers have explored the optimal control, especially the linear quadratic regulator (LQR), to realize the natural gait [28, 29, 30, 31]. The LQR scheme with full-state feedback yields control measures concerning the whole body compared to PD control for every independent joint [28]. In addition to that, the relative prominence of curtailing the tracking error and minimalizing the control torque can be regulated by computing optimal values of time-varying gain based on the design parameters of a single controller. Furthermore, LQR as a linear control scheme might be exploited for nonlinear system dynamics by approximating the linear time-varying form and significantly mitigating the computational complexity involved in several nonlinear controllers. Ajjanaromvat and Parnichkun [29] proposed an iterative online learning-based LQR control scheme for a treadmill-appended exoskeleton to investigate the robustness analysis. Moreover, the proposed control scheme is aided with an adaptive iterative learning control to address tracking errors. Gupta et al. [30] presented the LQR control for lower limb exoskeleton systems by considering the 4-DOF human gait model in the Single Support Phase (SSP). They exploited the nondominated sorting genetic algorithm to find out the optimal weighing matrix. However, the formulation work has not considered the uncertain factors in system dynamics. Castro et al. [31] proposed an integral-aided LQR (LQRi) and unknown input disturbance observer (UIO) to address external interferences of the lower limb exoskeleton system. The results of the proposed control are compared with proportional-derivative control and found to be more effective.

Although the hybrid form of sliding mode control can be considered a highly robust control strategy, chattering always affects the performance of exoskeleton systems. On the other hand, the LQR is the most optimal control scheme and lacks to resolve uncertain exoskeleton dynamics. Therefore, in this work, a new robust LQR-based neural-fuzzy control scheme is designed for the lower limb exoskeleton system with parametric uncertainties and external disturbances during passive gait rehabilitation training. The key highlights of the present work are as follows:

- The input-output feedback linearization approach is represented to linearize the nonlinear dynamics of the lower limb exoskeleton system
- A robust offline LQR-based neural-fuzzy control scheme is designed to deal with payload uncertainties
- A disturbance estimator is proposed using an online adaptation of firing strength in offline designed LQR-NF architecture
- The simulation results are carried out for the RLQR-NF control scheme and compared with an exponential reaching law-based sliding mode control (ERL-SM) to track the desired gait trajectory during passive therapeutic training
- The robustness performance of the proposed control scheme (RLQR-NF) is investigated by varying payload parameters and inducing different forms of external disturbances

The rest of the paperwork is structured as follows. The mechanical description of the lower limb exoskeleton system and the estimation of control input parameters are presented in Section 2. In Section 3, the nonlinear dynamic relation is formulated using the Euler-Lagrange principle, and thereafter, input-output linearization of the nonlinear form is explained.  Section 4 presents the concept of ANFIS architecture with the selected membership function.  Section 5 describes a detailed design procedure of the proposed control strategy. In Section 6, the Lyapunov theory of stability is presented. The control results are simulated and discussed in Section 7. The complete paperwork is concluded in Section 8.

## 2. Mechanical Configuration of the Lower Limb Exoskeleton System

The main criteria for the mechanical design of a lower limb exoskeleton system are to ensure its strength and stability of the subject's safety. Moreover, the adaptability of the system with different heights of the subjects augments the feature of cost-effectiveness. Considering the subject's physiological safety, all possible degrees of freedom should be avoided at the initial phases of rehabilitation training. Invoking the design features, authors have designed a low-cost stand-alone module-aided lower limb exoskeleton system for pediatric rehabilitation in their previous work [32]. The CAD model of the designed exoskeleton system is shown in Figures 1(a) and 1(b). A 3-DOF multilink mechanism for each leg was intended to carry out hip flexion/extension, knee flexion/extension, and ankle dorsiflexion/plantarflexion motions. The placements of the joint actuators were made to avoid any physical interference with the subject's body. To serve subjects of different heights, a telescopic link joint arrangement was designed around the knee joint of the exoskeleton system. Moreover, a detailed structural analysis of the stand-alone module was carried for maximum loading conditions at the hip joint [32].

The mechanical configuration of the exoskeleton system is intended for children of 8-12 years of age, 25-40 kg weight, and 115-125 cm height. The possible range of motion (ROM) for three joints of the exoskeleton system in the sagittal plane is as follows: 30°/-12° (hip-f/e), 60°/-10° (knee-f/e), and 13°/-20° (ankle-d/p). To avoid any undesirable actions beyond the ROM, an emergency stop option is provisioned at the software interface during simulation runs. In this work, an eight-year-old male subject's anthropometric and kinematic parameters (body mass: 30 kg and body height: 1.22 m) are considered input parameters to the control architecture. The breakdown of input parameters for the lower limb exoskeleton and subject is shown in Table 1, where the length of the thigh and shank link is kept constant at 0.27 m and 0.30 m, respectively.

Furthermore, an affordable wireless Labview-aided Kinect setup was established to conduct the experimental gait analysis. With necessary approval, the child subject was asked to follow an inclined path over the ground in front of the experimental setup for 1.6-2.0 seconds. The angle estimation algorithm comprehended the information about the lower limb joint angles from the skeleton model in Labview. The angle estimation algorithm exploits the relation between joint triples using vector algebra.

The detailed procedure of performing gait analysis, as shown in Figure 2(a), is based on the work by Narayan et al. [33]. The skeleton form of the subject during the gait analysis is illustrated in Figure 2(b). The desired lower limb joint angles attained from the experiment are presented in Figure 3(a) and the corresponding trajectory in Figure 3(b). The ROM for the hip, knee, and ankle joints are recorded as 22.16° to -8.98°, 58.26° to 1.21°, and 5.84° to -7.94° for an eight-year-old child, respectively.

## 3. Dynamic Model of the Coupled Human-Exoskeleton System

In this section, the Euler-Lagrange principle is used to formulate the nonlinear dynamics of the coupled human-exoskeleton system. Thereafter, the input-output feedback linearization approach is exploited to linearize the nonlinear behavior of the dynamical system. The transformed linear state-space relation is established for the dynamics of the lower limb exoskeleton system.

### 3.1. Nonlinear Dynamic Formulation

Among various methods for expressing applied joint torques and angular acceleration, the Euler-Lagrange principle is well appreciated by the research communities [34]. Invoking the Euler-Lagrange principle, which employs kinetic and potential energy, the nonlinear representation of the coupled human-exoskeleton dynamics is obtained. A multilink structure of the coupled system with a collaboration effect is shown in Figures 4(a) and 4(b).

A generalized formulation to estimate the joint torques using the Lagrangian *L* is as follows:

(1) $$\begin{array}{c} \tau =\frac{d}{dt}\left(\frac{\partial L}{\partial {\dot{\theta }}_{i}}\right)-\frac{\partial L}{{\partial \theta }_{i}}, \end{array}$$

(2) $$\begin{array}{c} L=K-P, \end{array}$$

where

(3) $$\begin{array}{c} K=\overset{3}{\underset{i=1}{\sum }}\left(\frac{1}{2}m_{i}{\dot{s}}_{i}^{T}{\dot{s}}_{i}+\frac{1}{2}{\dot{\theta }}_{i}^{T}I_{i}{\dot{\theta }}_{i}\right), \end{array}$$

(4) $$\begin{array}{c} P=\overset{3}{\underset{i=1}{\sum }}\left(m_{i}gh_{\text{c}i}\right). \end{array}$$

In the abovementioned relations, *θ*_*i*_ represents the generalized coordinate of the human-exoskeleton system. The kinetic and potential energy about the *i*-link is denoted by *K* and *P*, respectively. In Equation (3), ${\dot{\theta }}_{i}$, ${\dot{s}}_{i}$, *m*_*i*_, and *I*_*i*_ signify the angular velocity, speed of the center of mass in translational direction, mass, and inertia corresponding to the *i*-link. The acceleration due to the gravitational effects is referred by *g*, and the distance between the *i*-link's center point forming the gravitational vector and the origin is denoted by *h*_c*i*_ as illustrated in Equation (4).

Referring to Equations (2)–(4) to solve Equation (1), the nonlinear dynamics of the coupled dynamical system can be articulated as follows:

(5) $$\begin{array}{c} \tau =M\left(\theta \right)\ddot{\theta }+C\left(\theta ,\dot{\theta }\right)\dot{\theta }+G\left(\theta \right), \end{array}$$

where

(6) $$\begin{array}{c} \left\{\begin{array}{c} \tau =\tau_{\text{a}}+\tau_{\text{eh}}+\tau_{\text{he}},\\ M\left(\theta \right)=M^{\text{e}}\left(\theta \right)+M^{\text{h}}\left(\theta \right),\\ C\left(\theta ,\dot{\theta }\right)=C^{\text{e}}\left(\theta ,\dot{\theta }\right)+C^{\text{h}}\left(\theta ,\dot{\theta }\right),\\ G\left(\theta \right)=G^{\text{e}}\left(\theta \right)+G^{\text{h}}\left(\theta \right), \end{array}\right. \end{array}$$

(7) $$\begin{array}{c} M\left(\theta \right)=\left[\begin{array}{ccc} M_{11} & M_{12} & M_{13}\\ M_{21} & M_{22} & M_{23}\\ M_{31} & M_{32} & M_{33} \end{array}\right], \end{array}$$

The matrix form of inertial, Coriolis-centrifugal, and gravity effects of the coupled dynamical system is signified by *M*(*θ*), $C\left(\theta ,\dot{\theta }\right)$, and *G*(*θ*), respectively. In Equation (6), *M*^e^(*θ*) and *M*^h^(*θ*) represent the inertial dynamics of the exoskeleton and human leg in the matrix form, respectively. The Coriolis-centrifugal matrix of the exoskeleton and human leg is represented by $C^{\text{e}}\left(\theta ,\dot{\theta }\right)$, and $C^{\text{h}}\left(\theta ,\dot{\theta }\right)$, respectively. The gravity matrix of the exoskeleton and human leg is referred by *G*^e^(*θ*) and *G*^h^(*θ*), respectively.  *τ*_a_ implies the actuator torque while driving the joint of a human's lower limb. The collaboration torque is indicated by *τ*_eh_ and *τ*_he_ for collaboration of exoskeletons with humans and vice versa, respectively.

During exoskeleton-human interaction, splints are exploited to keep the exoskeleton link and human leg attached, which induces the collaboration torques (*τ*_eh_ and *τ*_he_). However, in passive gait rehabilitation, as considered in the present work, these collaborations are withdrawn by assuming rigid connections and matching joint angles for exoskeletons and humans. As illustrated in Figure 4(b), the interaction dynamics is formulated as below:

(8) $$\begin{array}{c} \tau_{\text{eh}}=-\tau_{\text{he}}=J^{T}f_{\text{co}}=J^{T}\left(k\Delta x+c\Delta \dot{x}\right)=k\left(\theta_{\text{h}}-\theta_{\text{e}}\right)+c\left({\dot{\theta }}_{\text{h}}-{\dot{\theta }}_{\text{e}}\right), \end{array}$$

where *f*_co_ represents the collaboration force between the exoskeleton and the human, *k* and *c* signify the mechanical stiffness and damping factors of the used splints, Δ*x* denotes the Cartesian coordinate disparity between the human leg and the exoskeleton link, and (*θ*_h_ − *θ*_e_) refers to the joint angular disparity between the human leg and the exoskeleton link.

Furthermore, in the presence of parametric uncertainties and external disturbances, Equation (5) can be rewritten as

(9) $$\begin{array}{c} \overset{ˇ}{\tau }=\overset{ˇ}{M}\left(\theta \right)\ddot{\theta }+\overset{ˇ}{C}\left(\theta ,\dot{\theta }\right)\dot{\theta }+\overset{ˇ}{G}\left(\theta \right), \end{array}$$

where

(10) $$\begin{array}{c} \left\{\begin{array}{c} \overset{ˇ}{\tau }=\eta \;\tau +D,\\ \overset{ˇ}{M}\left(\theta \right)=M\left(\theta \right)+\eta \;M\left(\theta \right),\\ \overset{ˇ}{C}\left(\theta ,\dot{\theta }\right)=C\left(\theta ,\dot{\theta }\right)+\eta \;C\left(\theta ,\dot{\theta }\right),\\ \overset{ˇ}{G}\left(\theta \right)=G\left(\theta \right)+\eta \;G\left(\theta \right), \end{array}\right. \end{array}$$

where *D* denotes the external disturbances applied by the subjects to the system; *η* is the uncertain scaling factor when considering the same amount of variation in dynamic parameters.

After considering joint torques (*τ*) equivalent to joint actuator torques (*τ*_a_) in case of passive rehabilitation training, the actuator dynamics can be formulated using Kirchhoff's law to obtain the control voltage (${\overset{ˇ}{U}}_{m}$) as follows:

(11) $$\begin{array}{c} {\overset{ˇ}{U}}_{m}=\frac{\overset{ˇ}{\tau }\;R_{m}}{S_{m}}+{\dot{i}}_{m}L_{m}+\Xi_{e}\dot{\theta }, \end{array}$$

where *R*_*m*_, *S*_*m*_, ${\dot{i}}_{m}$, *L*_*m*_, and *Ξ*_*e*_ denote the armature resistance, torque sensitivity, current, armature inductance, and back EMF constant of the DC motor. These parameters are selected from the specification sheet provided by Bholanath Precision Engineering Private Limited [35].

To imitate the realistic cases, the actuator saturation should be considered in the design of the control law to avoid the hysteresis cycle and maintain the linearity of the actuator. Moreover, this ensures closed-loop stability by limiting the large control signals. Based on the saturation theory, the control signal $\left({\overset{ˇ}{U}}_{m}\right)$ from Equation (11) can be further defined as below:

(12) $$\begin{array}{c} {\overset{ˇ}{U}}_{m}=\left\{\;\begin{array}{c} {℧}_{m}\;\left({\overset{ˇ}{U}}_{m}>{℧}_{m}\right),\\ {\overset{ˇ}{U}}_{m}\;\left(\left|{\overset{ˇ}{U}}_{m}\right|\leq {℧}_{m}\right),\\ -{℧}_{m}\;\;\left({\overset{ˇ}{U}}_{m}<{-℧}_{m}\right), \end{array}\right. \end{array}$$

where ℧∈ℝ^3^ denotes a vector with positive elements. The upper and lower saturation bound is denoted by ℧_*m*_ and −℧_*m*_, respectively.

### 3.2. Input-Output Feedback Linearization

The main objective of the feedback linearization is to correctly linearize the nonlinear dynamics with suitable modifications in state-space coordinates using an inner loop control [34]. Thereafter, an outer loop control with a new set of coordinates can be formed to establish a linear relationship between the output vector (*y*) and the input vector ($\overset{ˇ}{u}$) and validate the cost functions of the control design. Consider the nonlinear multiple-input and single-output (MISO) dynamic relation with *n* as the order and *p* as the total number of inputs as well as outputs, defined in the affine state:

(13) $$\begin{array}{c} \left\{\begin{array}{c} \dot{x}\left(t\right)=\Psi \left(x\left(t\right)\right)+\overset{p}{\underset{i=1}{\sum }}\Pi_{i}\left(x\left(t\right)\right){\overset{ˇ}{U}}_{m_{i}}\left(t\right),\\ y_{i}\left(t\right)=\Lambda_{i}\left(x\left(t\right)\right), \end{array}\right. \end{array}$$

where *x* = [*𝓍*_1_, *𝓍*_2_, ⋯,*𝓍*_*n*_]^*T*^ ∈ ℝ^*n*^ denotes the state vector, ${\overset{ˇ}{U}}_{m_{i}}={\left[{\overset{ˇ}{U}}_{m_{1}},{\overset{ˇ}{U}}_{m_{2}},\cdots ,{\overset{ˇ}{U}}_{m_{p}}\right]}^{T}\in {\mathbb{R}}^{p}$ signifies the control input vector, and *y* = [*𝓎*_1_, *𝓎*_2_, ⋯,*𝓎*_*p*_]^*T*^ ∈ ℝ^*p*^ indicates the output vector.

**Theorem 1 .**

Suppose Ψ : ℝ^*n*^⇒ℝ^*n*^ signifies a smooth vector field on ℝ^*n*^ and *Λ* : ℝ^*n*^⇒ℝ^*n*^ denotes a scalar function. Then, the Lie derivative of *Λ* to Ψ, referred as *L*_Ψ_*Λ*, is expressed as follows [36, 37]:

(14) $$\begin{array}{c} L_{\Psi }\Lambda =\frac{\partial \Lambda }{\partial x}\Psi \left(x\right)=\overset{p}{\underset{i=1}{\sum }}\frac{\partial \Lambda }{\partial x_{i}}\Psi \left(x\right). \end{array}$$

Similarly, the Lie derivative of *L*_Ψ_*Λ* with respect to Ψ is defined as

(15) $$\begin{array}{c} L_{\Psi }^{2}\;\Lambda =L_{\Psi }\;\left(L_{\Psi }\Lambda \right). \end{array}$$

In general,

(16) $$\begin{array}{c} L_{\Psi }^{\gamma }\;\Lambda =L_{\Psi }\left(L_{\Psi }^{\gamma -1}\;\Lambda \right)\;\text{with }L_{\Psi }^{0}\;\Lambda =\Lambda ,\forall \gamma =1,\cdots ,p. \end{array}$$

**Theorem 2 .**

The function **Φ** : ℝ^*n*^⇒ℝ^*n*^, specified in a region *Y* ⊂ ℝ^*n*^, is termed as diffeomorphism if the function **Φ** along with the inverse **Φ**^−1^ (if it exists) is smooth, i.e., differentiable everywhere [36, 37].

However, as the global diffeomorphism is rare, one should check for local diffeomorphisms, i.e., transformations defined in a limited neighborhood of a specified point [37]. With the concept of diffeomorphism, we transform a nonlinear system into another one by changing the variables in the following form:

(17) $$\begin{array}{c} z={\left[z_{1},z_{2},\cdots ,z_{n}\right]}^{T}=\Phi \left(x\right), \end{array}$$

where **Φ**(*x*) characterizes *n* variables as

(18) $$\begin{array}{c} \Phi \left(x\right)=\left[\begin{array}{c} \begin{array}{c} \Phi_{1}\\ \Phi_{2}\\ \vdots \end{array}\\ \Phi_{n} \end{array}\right]=\left[\begin{array}{c} {\left[\Lambda_{1}\;L_{\Psi }\Lambda_{1}\;\cdots \;L_{\Psi }^{r_{1}-1}\Lambda_{1}\right]}^{T}\\ \vdots \\ {\left[\Lambda_{p}\;L_{\Psi }\Lambda_{p}\;\cdots \;L_{\Psi }^{r_{p}-1}\Lambda_{p}\right]}^{T} \end{array}\right], \end{array}$$

with *x* = [*𝓍*_1_, *𝓍*_2_, ⋯,*𝓍*_*n*_]^*T*^.

Now, a linear relationship between inputs and outputs is to be established by performing the differentiation of the outputs (*𝓎*_*i*_) till the input terms appear in the formulation. Considering *r*_*j*_ is the smallest integer, (*𝓎*_*j*_^(*r*_*j*_)^) can be evaluated with a complete term of inputs as follows:

(19) $$\begin{array}{c} y_{j}^{\left(r_{j}\right)}=L_{\Psi }^{r_{j}}\Lambda_{j}\left(x\right)+\overset{p}{\underset{i=1}{\sum }}L_{\Pi_{i}}\left(L_{\Psi }^{r_{j-1}}\Lambda_{j}\left(x\right)\right){\overset{ˇ}{U}}_{m_{i}},\;i,j=1,2,\cdots ,p, \end{array}$$

where *L*_Ψ_^*i*^*Λ*_*j*_ and *L*_**Π**_^*i*^*Λ*_*j*_ signify the *i*th Lie derivatives of *Λ*_*j*_(*x*) in the direction of Ψ and **Π**, respectively. In Equation (19), *r*_*j*_ denotes the relative degree for the output *𝓎*_*j*_ which provides information about the number of derivatives required to carry out at least one of the inputs in the formulation [37, 38]. The sum of every relative degree from Equation (19) constitutes the total relative degree (*r*) which needs to be less than or equal to the system's order.

(20) $$\begin{array}{c} r=\overset{n}{\underset{j=1}{\sum }}r_{j}\leq n. \end{array}$$

Furthermore, rewriting Equation (19) and expressing the nonlinear control law ${\overset{ˇ}{U}}_{m}$ to form the linear relationship between the input and the output as follows, one can get

(21) $$\begin{array}{c} {\left[y_{1}^{r_{1}},\cdots ,y_{p}^{r_{p}}\right]}^{T}=\delta \left(x\right)+\sigma \left(x\right)\cdot {\overset{ˇ}{U}}_{m}, \end{array}$$

(22) $$\begin{array}{c} \overset{ˇ}{u}={\left[{\overset{ˇ}{u}}_{1},{\overset{ˇ}{u}}_{2},\cdots ,{\overset{ˇ}{u}}_{p}\right]}^{T}={\left[y_{1}^{r_{1}},\cdots ,y_{p}^{r_{p}}\right]}^{T}, \end{array}$$

where

(23) $$\begin{array}{c} \left\{\begin{array}{c} \delta \left(x\right)=\left[\begin{array}{c} \begin{array}{c} L_{\Psi }^{r_{1}}\Lambda_{1}\left(x\right)\\ \vdots \\ \vdots \end{array}\\ L_{\Psi }^{r_{p}}\Lambda_{p}\left(x\right) \end{array}\right],\\ \sigma \left(x\right)=\left[\begin{array}{c} L_{\Pi_{1}}\left(L_{\Psi }^{\left(r_{1-1}\right)}\Lambda_{1}\left(x\right)\right)L_{\Pi_{2}}\left(L_{\Psi }^{\left(r_{1}-1\right)}\Lambda_{1}\left(x\right)\right)\cdots L_{\Pi_{p}}\left(L_{\Psi }^{\left(r_{1}-1\right)}\Lambda_{1}\left(x\right)\right)\\ L_{\Pi_{1}}\left(L_{\Psi }^{\left(r_{2}-1\right)}\Lambda_{2}\left(x\right)\right)L_{\Pi_{2}}\left(L_{\Psi }^{\left(r_{2}-1\right)}\Lambda_{2}\left(x\right)\right)\cdots L_{\Pi_{p}}\left(L_{\Psi }^{\left(r_{2}-1\right)}\Lambda_{2}\left(x\right)\right)\\ \vdots \;\vdots \;\vdots \\ L_{\Pi_{1}}\left(L_{\Psi }^{\left(r_{p}-1\right)}\Lambda_{p}\left(x\right)\right)L_{\Pi_{2}}\left(L_{\Psi }^{\left(r_{p-1}\right)}\Lambda_{p}\left(x\right)\right)\cdots L_{\Pi_{p}}\left(L_{\Psi }^{\left(r_{p}-1\right)}\Lambda_{p}\left(x\right)\right) \end{array}\right]. \end{array}\right. \end{array}$$

Assuming *σ*(*x*) is not singular, the input transferred form, i.e., the nonlinear control law, can be possibly defined as

(24) $$\begin{array}{c} {\overset{ˇ}{U}}_{m}=\sigma {\left(x\right)}^{-1}\left(-\delta \left(x\right)+\overset{ˇ}{u}\right), \end{array}$$

where $\overset{ˇ}{u}={\left[{\overset{ˇ}{𝓊}}_{1},{\overset{ˇ}{𝓊}}_{2},\cdots ,{\overset{ˇ}{𝓊}}_{p}\right]}^{T}$ and ${\overset{ˇ}{U}}_{m}={\left[{\overset{ˇ}{U}}_{m_{1}},{\overset{ˇ}{U}}_{m_{2}},\cdots ,{\overset{ˇ}{U}}_{m_{p}}\right]}^{T}$.

In Equation (24), $\overset{ˇ}{u}$ denotes the new input vector, ${\overset{ˇ}{U}}_{m}$ refers to the decoupling control law, *σ*(*x*) signifies an invertible matrix of order *p* × *p*, and *δ*(*x*) represents a decoupling matrix of the system.

Furthermore, the linearizing law from Equation (24) is applied for transforming the nonlinear dynamics of the coupled human-exoskeleton system (Equation (9)) into the linear state-space representation as follows:

(25) $$\begin{array}{c} \left\{\begin{array}{c} \dot{z}=\overset{ˇ}{A}z+\overset{ˇ}{B}\overset{ˇ}{u},\\ y=Cz, \end{array}\right. \end{array}$$

where $\overset{ˇ}{A}=A+\Delta A$, $\overset{ˇ}{B}=B+\Delta B$, and $\overset{ˇ}{u}=\left(\Delta +1\right)u+d$.

$\overset{ˇ}{A}$ and $\overset{ˇ}{B}$ are the state-weight factor matrices with the effect of parametric uncertainties; *A*, *B*, and *C* denote the state-weight factor matrices evaluated with nominal system parameters, i.e., in the absence of parametric uncertainties; Δ is the uncertain scaling factor in the linearized state-space form related to state-weight factor matrices and can be expressed in terms of dynamic parameters of the given system [39]. The input vector $\overset{ˇ}{u}$ carries the effect of parameter variations and external disturbances. The input vector in the absence of PUEDs is denoted by *u*. The disturbance applied to the system after feedback linearization is denoted by *d*, being analogous to *D* from Equation (9). The linearized dynamics in Equation (25) stands valid with the following assumptions:

*A1*: the $\left(\overset{ˇ}{A},\overset{ˇ}{B}\right)$ is in the controllable form.

*A2*: the disturbance *d* is in the bounded form.

In the present work, the state vector and output vector related to the hip, knee, and ankle joints of the coupled dynamical system is considered $z={\left[\theta_{H}\;\theta_{K}\;\theta_{A}\;{\dot{\theta }}_{H}\;{\dot{\theta }}_{K}\;{\dot{\theta }}_{A}\right]}^{T}$ and *y* = [*θ*_*H*_ *θ*_*K*_ *θ*_*A*_]^*T*^, respectively. The input vector with nominal system parameters is defined as *u* = [*u*_*H*_ *u*_*K*_ *u*_*A*_]^*T*^. Moreover, the respective state-weight factor matrices (*A* ∈ ℝ^6×6^, *B* ∈ ℝ^6×3^, and *C* ∈ ℝ^3×6^) can be formulated as below. The entries of these matrices are extensively presented in the appendix.

(26) $$\begin{array}{c} \left\{\begin{array}{c} A={\left(\begin{array}{cc} {\left[0\right]}_{3\times 3} & I_{3}\\ \begin{array}{ccc} \frac{\alpha_{41}}{{\tilde{\alpha }}_{41}} & \frac{\alpha_{42}}{{\tilde{\alpha }}_{42}} & \frac{\alpha_{43}}{{\tilde{\alpha }}_{43}}\\ \frac{\alpha_{51}}{{\tilde{\alpha }}_{51}}-\frac{\alpha_{51^{\prime }}}{{\tilde{\alpha }}_{51^{\prime }}}+\frac{\alpha_{51^{\prime \prime }}}{{\tilde{\alpha }}_{51^{\prime \prime }}} & \frac{\alpha_{52}}{{\tilde{\alpha }}_{52}}-\frac{\alpha_{52^{\prime }}}{{\tilde{\alpha }}_{52^{\prime }}}+\frac{\alpha_{52^{\prime \prime }}}{{\tilde{\alpha }}_{52^{\prime \prime }}} & \frac{\alpha_{53}}{{\tilde{\alpha }}_{53}}+\frac{\alpha_{53^{\prime }}}{{\tilde{\alpha }}_{53^{\prime }}}-\frac{\alpha_{53^{\prime \prime }}}{{\tilde{\alpha }}_{53^{\prime \prime }}}\\ \frac{\alpha_{61}}{{\tilde{\alpha }}_{61}}-\frac{\alpha_{61^{\prime }}}{{\tilde{\alpha }}_{61^{\prime }}}-\frac{\alpha_{61^{\prime \prime }}}{{\tilde{\alpha }}_{61^{\prime \prime }}} & \frac{\alpha_{62}}{{\tilde{\alpha }}_{62}}-\frac{\alpha_{62^{\prime }}}{{\tilde{\alpha }}_{62^{\prime }}}-\frac{\alpha_{62^{\prime \prime }}}{{\tilde{\alpha }}_{62^{\prime \prime }}} & \frac{\alpha_{63}}{{\tilde{\alpha }}_{63}}-\frac{\alpha_{63^{\prime }}}{{\tilde{\alpha }}_{63^{\prime }}}-\frac{\alpha_{63^{\prime \prime }}}{{\tilde{\alpha }}_{63^{\prime \prime }}} \end{array} & {\left[0\right]}_{3\times 3} \end{array}\right)}_{6\times 6},\\ B={\left(\begin{array}{c} {\left[0\right]}_{3\times 3}\\ \begin{array}{ccc} \frac{\beta_{41}}{{\tilde{\beta }}_{41}} & \frac{\beta_{42}}{{\tilde{\beta }}_{42}} & \frac{\beta_{43}}{{\tilde{\beta }}_{43}}\\ \frac{\beta_{51}}{{\tilde{\beta }}_{51}} & \frac{\beta_{52}}{{\tilde{\beta }}_{52}} & \frac{\beta_{53}}{{\tilde{\beta }}_{53}}\\ \frac{\beta_{61}}{{\tilde{\beta }}_{61}} & \frac{\beta_{62}}{{\tilde{\beta }}_{62}} & \frac{\beta_{63}}{{\tilde{\beta }}_{63}} \end{array} \end{array}\right)}_{6\times 3},\\ C={\left(\begin{array}{c} 1\\ 0\\ 0 \end{array}\;\begin{array}{c} 0\\ 1\\ 0 \end{array}\;\begin{array}{c} 0\\ 0\\ 1 \end{array}\;\begin{array}{c} 0\\ 0\\ 0 \end{array}\;\begin{array}{c} 0\\ 0\\ 0 \end{array}\;\begin{array}{c} 0\\ 0\\ 0 \end{array}\right)}_{3\times 6}. \end{array}\right. \end{array}$$

## 4. Adaptive Neural-Fuzzy Inference System

The adaptive neural-fuzzy inference system (ANFIS), colloquially known as the neural-fuzzy or neuro-fuzzy (NF) system, was proposed by Jang and Sun [40] by augmenting the benefits of adaptive neural networks and fuzzy reasoning. In the NF system, IF-THEN-based fuzzy logic inferences are constructed to form the learning rules with a defined input-output dataset and reproduce the output vector with zero error tolerance. A neural-fuzzy system exploits the fuzzy input variables and input-dependent nonfuzzy output variables given by Takagi and Sugeno [41]. For instance,

If the acceleration of the robot′s end − effector is *high*, then

(27) $$\begin{array}{c} f\left(t\right)=c\times {\left(\text{acceleration of the robo}{\text{t}}^{\text{'}}\text{s end}-\text{effector}\right)}^{2}. \end{array}$$

In Equation (27), *high* signifies a fuzzy label with the membership function (MF), representing the acceleration of the robot′s end − effector in the rule proposition. The rule subsequent with nonfuzzy behavior is formulated according to the input variable of the premise step, acceleration of the robot′s end − effector.

### 4.1. ANFIS Architecture

A neural-fuzzy system inherently exploits the five layers. The primary network architecture with two input vectors (*𝓏* : *x*, *y*) and one output vector (*f*(*𝓏*)) is considered to show the generalized process of ANFIS. As shown in Figure 5, two kinds of nodes are employed in the architecture: first, a square node for adaptation of the parameters, and second, a circular node that behaves as a fixed node with no parameter. The layer-by-layer development of the ANFIS structure is given below [42, 43].

**Layer 1 .**

This layer acts as a conversion function for the crisp value of the input vector into an appropriate MF-based fuzzy language, depicted as follows:

(28) $$\begin{array}{c} O_{j}^{1}=\Omega_{A_{j}}\left(x\right),\\ O_{j}^{1}=\Omega_{B_{j}}\left(y\right), \end{array}$$

where *𝒪*_*j*_^1^ represents the *j*th node output for the first layer. *Ω*_*A*_*j*__(*x*) and *Ω*_*B*_*j*__(*y*) denote the membership weightage of respective input variables, defined for *A*_*j*_- and *B*_*j*_-type MF. In this work, the generalized bell membership function is chosen to replicate a proper probability distribution behavior and expressed as follows:

(29) $$\begin{array}{c} \text{bell}\left(z:a_{j},b_{j},c_{j}\right)=\Omega_{A_{j}}\left(x\right)=\Omega_{B_{j}}\left(y\right)=\frac{1}{1+{\left[{\left(\left(z-c_{j}\right)/a_{j}\right)}^{2}\right]}^{b_{j}}}. \end{array}$$

In Equation (29), “*a*_*j*_” and “*b*_*j*_” signify the width and shape parameters of the membership function. The value of “*b*_*j*_” is generally positive; however, it can be considered negative in case of inverted shape. “*c*_*j*_” indicates the center position of the membership function. Having an extra parameter compared to Gaussian MF, the generalized bell has the added advantage of tuning the steepness at crossover positions.

**Layer 2 .**

This layer evaluates the firing strength for every rule using a product of incoming signals from each circular node. It is designated by notation **Π** in the ANFIS architecture. The following expression is used to estimate the firing strength (*w*_*j*_) as follows:

(30) $$\begin{array}{c} O_{j}^{2}=w_{j}=\Omega_{A_{j}}\left(x\right)=\Omega_{B_{j}}\left(y\right),\;j=1,2. \end{array}$$

**Layer 3 .**

In this layer, the normalization of the node's firing strength is carried out by dividing the *j*th rule firing strength to all rules' total firing strength. This layer is designated by notation *N* in the ANFIS architecture. The firing strength (${\bar{w}}_{j}$) is normalized as follows:

(31) $$\begin{array}{c} O_{j}^{3}={\bar{w}}_{j}=\frac{w_{j}}{w_{1}+w_{2}},\;j=1,2. \end{array}$$

**Layer 4 .**

This layer, having the square nodes, is used to estimate the rule's involvement by defuzzification of input variables and produce the respective output as follows:

(32) $$\begin{array}{c} O_{j}^{4}={\bar{w}}_{j}{∠}_{j}={\bar{w}}_{j}\left(p_{j}x+q_{j}y+r_{j}\right), \end{array}$$

where ${\bar{w}}_{j}$ indicates the normalized firing strength and *p*_*j*_, *q*_*j*_, and *r*_*j*_ signify the subsequent limits.

**Layer 5 .**

This layer, having circular shape nodes with the designation ∑, processes the final output using the summation of all incoming signals from the preceding layer. Mathematically, it can be expressed as follows:

(33) $$\begin{array}{c} O_{j}^{5}=\underset{j}{\sum }{\bar{w}}_{j}{∠}_{j}=\frac{\sum_{j}w_{j}{∠}_{j}}{\sum_{j}w_{j}}. \end{array}$$

## 5. Robust Design of the LQR-Based Neural-Fuzzy Control

The design procedure of RLQR-NF control is organized into two parts: first, the offline training of a robust LQR-based ANFIS training dataset to deal with parametric uncertainties, and second, the online training of the LQR-based ANFIS architecture using the adaptive law of weights to compensate for the external disturbances. In both parts, the effects of parametric uncertainties and external disturbances are explicitly considered. Thereafter, the stability of the proposed control strategy in the presence of PUEDs is addressed by the Lyapunov theory in the next section.

### 5.1. Offline Training of the RLQR-NF Dataset for Parametric Uncertainties

As shown in Figure 6, this subsection is further presented into two stages: first, the formulation of a robust LQR-NF dataset by varying mass parameters, and second, the stepwise layout of offline training of a dataset using ANFIS parameters to design the robust control strategy.

#### 5.1.1. Stage I: Formulation of the RLQR-NF Training Dataset

The training dataset, having multiple-input and single-output (MISO), is formed by employing the concepts of the LQR control strategy as shown in Equation (25). The LQR cost function is considered a minimization problem while applying the optimality conditions and is expressed as follows [44]:

(34) $$\begin{array}{c} J=\frac{1}{2}\int_{0}^{\infty }\left(z^{T}Qz+{\overset{ˇ}{u}}^{T}R\overset{ˇ}{u}\right)dt, \end{array}$$

where *Q* and **R** denote the user-defined state-weight matrix and control cost matrix, respectively. An appropriate selection of both matrices directly influences the performance characteristics of the controller.

The generalized input ($\overset{ˇ}{u}$) to the control system is articulated by regulating the error vector (**ℯ**) as follows:

(35) $$\begin{array}{c} \overset{ˇ}{u}=Kℯ=K\left(z_{\text{des}}-z\right), \end{array}$$

where *z*_des_ and *z* represent the desired and actual state vectors, respectively. The optimal state gain matrix (*K*) can be expressed in terms of the control cost matrix (**R**) and the state-weight factor matrix ($\overset{ˇ}{B}$) as follows:

(36) $$\begin{array}{c} K=R^{-1}{\overset{ˇ}{B}}^{T}P, \end{array}$$

where *P* is the answer for the algebraic form of the Riccati equation expressed in the form of state-weight factor matrices ($\overset{ˇ}{A}$ and $\overset{ˇ}{B}$), state-weight matrix (*Q*), and control cost matrix (**R**) as given below [44, 45]:

(37) $$\begin{array}{c} P\overset{ˇ}{A}+{\overset{ˇ}{A}}^{T}P-P\overset{ˇ}{B}R^{-1}{\overset{ˇ}{B}}^{T}P+Q=0. \end{array}$$

It is truly evident from Equation (36) that the state gain matrix (*K*) is regulated by $\overset{ˇ}{A}$, $\overset{ˇ}{B}$, *Q*, and **R** matrices where $\overset{ˇ}{A}$ and $\overset{ˇ}{B}$ are reliant on the mechanical arrangement and dynamic parameters of the requisite system.

Exploiting the controller's gain (*K*), a generalized dataset (*S*_*d*_) with the error vector (**ℯ**) and respective input ($\overset{ˇ}{u}$) to the control system can be created in the following form [44]:

(38) $$\begin{array}{c} S_{d}=\left[{ℯ}^{T}\;\overset{ˇ}{u}\right]. \end{array}$$

In this work, the dataset (*S*_*d*_) is expanded into a robust form by evaluating the controller's gain (*K*_*m*_t_,*m*_c_,*m*_hf__) for a bounded variation of the coupled thigh (*m*_t_), calf (*m*_c_), and heel-foot (*m*_hf_) masses of the human-exoskeleton system. Thereafter, the controller input $\left({\overset{ˇ}{u}}_{m_{\text{t}},m_{\text{c}},m_{\text{hf}}}\right)$ for the hip, knee, and ankle joints is formulated as follows:

(39) $$\begin{array}{c} {\overset{ˇ}{u}}_{m_{\text{t}},m_{\text{c}},m_{\text{hf}}}=K_{m_{\text{t}},m_{\text{c}},m_{\text{hf}}}ℯ, \end{array}$$

where

(40) $$\begin{array}{c} {\overset{ˇ}{u}}_{m_{\text{t}},m_{\text{c}},m_{\text{hf}}}={\left[{\overset{ˇ}{u}}_{{\text{H}}_{m_{\text{t}},m_{\text{c}},m_{\text{hf}}}}\;{\overset{ˇ}{u}}_{{\text{K}}_{m_{\text{t}},m_{\text{c}},m_{\text{hf}}}}\;{\overset{ˇ}{u}}_{{\text{A}}_{m_{\text{t}},m_{\text{c}},m_{\text{hf}}}}\right]}^{T}, \end{array}$$

(41) $$\begin{array}{c} ℯ={\left[{ℯ}_{\theta_{\text{H}}}\;{ℯ}_{\theta_{\text{K}}}\;{ℯ}_{\theta_{\text{A}}}\;{ℯ}_{{\dot{\theta }}_{\text{H}}}\;{ℯ}_{{\dot{\theta }}_{\text{K}}}\;{ℯ}_{{\dot{\theta }}_{\text{A}}}\right]}^{T}. \end{array}$$

In Equation (40), ${\overset{ˇ}{u}}_{{\text{H}}_{m_{\text{t}},m_{\text{c}},m_{\text{hf}}}}$, ${\overset{ˇ}{u}}_{{\text{K}}_{m_{\text{t}},m_{\text{c}},m_{\text{hf}}}}$, and ${\overset{ˇ}{u}}_{{\text{A}}_{m_{\text{t}},m_{\text{c}},m_{\text{hf}}}}$ denote the controller output for the hip, knee, and ankle joints of the exoskeleton device, respectively. In Equation (41), **ℯ**_*θ*_H__, **ℯ**_*θ*_K__, and **ℯ**_*θ*_A__ signify the hip, knee, and ankle joint angular errors, respectively. ${ℯ}_{{\dot{\theta }}_{\text{H}}}$, $\;{ℯ}_{{\dot{\theta }}_{\text{K}}}$, and ${ℯ}_{{\dot{\theta }}_{\text{A}}}$ represent the respective errors of the hip, knee, and ankle joint angular velocities.

The expanded structure of the robust dataset (*S*_rd_) is finally depicted as below:

(42) $$\begin{array}{c} S_{\text{rd}}=\left[{ℯ}^{T}\;{\overset{ˇ}{u}}_{m_{\text{t}},m_{\text{c}},m_{\text{hf}}}\right], \end{array}$$

where

(43) $$\begin{array}{c} S_{\text{rd}}={\left[S{\left(1\right)}_{\text{rd}}\;S{\left(2\right)}_{\text{rd}}\;S{\left(3\right)}_{\text{rd}}\right]}^{T}. \end{array}$$

#### 5.1.2. Stage II: Stepwise Layout of Offline Training of the RLQR-NF Dataset

The layout and execution of the proposed control strategy for the exoskeleton device are presented in the following steps.

**Step 1 .**

The state gain matrix (*K*_*m*_t_,*m*_c_,*m*_hf__) is evaluated by solving Equations (36) and (37) for a different set of coupled thigh (*m*_t_), calf (*m*_c_), and heel-foot (*m*_hf_) masses, as shown in Table 2. The parametric variation is incorporated by increasing the nominal mass values up to 20%, with an increment of 0.3, 0.15, and 0.06 kg for the thigh, calf, and heel-foot. After performing several numerical experiments, the state-weight matrix and control cost matrix are selected as *Q* = diag(400000, 4000, 8000, 800, 8000, 800) and **R** = eye(3, 3).

**Step 2 .**

Apply Equation (39) to compute the controller input $\left({\overset{ˇ}{u}}_{m_{\text{t}},m_{\text{c}},m_{\text{hf}}}\right)$ for the operating range of state variables in the error vector as shown in Table 3. The structure of three robust datasets is formed by exploiting Equations (42) and (43).

**Step 3 .**

The training of robust datasets is carried out using the ANFIS approach. The first six columns of every dataset are inherently considered the input set. The last column of every dataset is regarded as the output set. The input set comprises the error vector (**ℯ**), and the output set contains the controller input vector $\left({\overset{ˇ}{u}}_{m_{\text{t}},m_{\text{c}},m_{\text{hf}}}\right)$. The three ANFIS architectures are formed, trained, and saved as *anfis1*.*fis*, *anfis2*.*fis*, and *anfis3*.*fis* for three controller inputs. Several simulation runs are performed by varying the number of MF from 1 to 50 and epochs from 1 to 30. Thereafter, the training parameters are selected based on the zero error tolerance between the desired and predicted output vectors. In general, ANFIS utilizes two optimization methods: backpropagation and hybrid, to establish the learning between the input and output vectors. A gradient descent model is employed to evaluate the node error in the backpropagation method. In contrast, a least square algorithm along with the gradient descent model is exploited to regulate the errors in the hybrid method. In this work, the hybrid method is used with all three datasets for training the neural-fuzzy networks. The complete details of training parameters are given in Table 4. After generating training files (*anfis1*.*fis*, *anfis2*.*fis*, and *anfis3*.*fis*) as the desired robust LQR-based neural-fuzzy controller, the respective signals are inputted to the nonlinear dynamics of the coupled human-exoskeleton system.

### 5.2. Online Training of the RLQR-NF Dataset for External Disturbances

Considering assumption A1, the control input with uncertain parameters $\left(\hat{u}\right)$ can be further expressed in terms of the state feedback (*Kz*) and disturbance observer $\left(\hat{d}\right)$ as

(44) $$\begin{array}{c} \hat{u}=\left(\Delta +1\right)u=\hat{d}-Kz, \end{array}$$

where $\hat{d}$ denotes the estimated disturbance by ANFIS architecture, and *K* signifies the state feedback matrix.

Substituting Equation (44) into Equation (22), the linearized dynamic model can be written as

(45) $$\begin{array}{c} \dot{z}=\left(\overset{ˇ}{A}-\overset{ˇ}{B}K\right)z+\overset{ˇ}{B}\;\left(\hat{d}+d\right). \end{array}$$

Now, the error dynamics of the control design in the time domain can be expressed as below:

(46) $$\begin{array}{c} \dot{ℯ}\left(t\right)=\left(\overset{ˇ}{A}-\overset{ˇ}{B}K\right)ℯ\left(t\right)+\overset{ˇ}{B}\;\left(\hat{d}\left(t\right)-f\left(t\right)\right), \end{array}$$

where

(47) $$\begin{array}{c} \overset{ˇ}{B}f\left(t\right)={\dot{z}}_{\text{des}}\left(t\right)-\overset{ˇ}{B}d\left(t\right)-\left(\overset{ˇ}{A}-\overset{ˇ}{B}K\right)z_{\text{des}}\left(t\right). \end{array}$$

Employing assumption A2, the *f*(*t*) can be considered a function with an upper limit. Therefore, the effectiveness of the coupled human-exoskeleton system can be augmented by estimating the *f*(*t*) from $\hat{d}\left(t\right)$. Using the ANFIS architecture mentioned in Section 4, the *f*(*t*) is approximated as follows [46, 47]:

(48) $$\begin{array}{c} f\left(z\right)={\overset{¯}{W}}^{T}\Omega \left(z\right)+\overset{¯}{\varrho }\left(z\right), \end{array}$$

where $\overset{¯}{W}$ denotes the ideal normalized firing strength matrix; **Ω**(*𝓏*) signifies the membership function vector; and $\overset{¯}{\varrho }\left(𝓏\right)$ represents an error of approximation with the condition $\overset{¯}{\varrho }\left(𝓏\right)\leq \zeta$, where *ζ* is a constant factor.

Now utilizing Equations (46) and (48), the error dynamics can be rewritten as

(49) $$\begin{array}{c} \dot{ℯ}\left(t\right)=\left(\overset{ˇ}{A}-\overset{ˇ}{B}K\right)ℯ\left(t\right)+\overset{ˇ}{B}\;\left(\hat{d}\left(t\right)-{\overset{¯}{W}}^{T}\Omega \left(z\right)-\overset{¯}{\varrho }\left(z\right)\right). \end{array}$$

From the above equation, the disturbance estimator $\hat{d}\left(t\right)$ is defined as follows to design the control law [47]:

(50) $$\begin{array}{c} {\hat{d}}_{i}={\hat{W}}_{ji}^{T}\Omega_{j}\left(z\right)-\zeta \mathrm{sign}\left({ℯ}^{T}P{\overset{ˇ}{B}}_{i}\right),\;i=1,2,\cdots ,p\text{ and }j=1,2,\cdots ,l, \end{array}$$

where *p* and *l* denote the number of inputs and network nodes in the hidden layer.

In the above expression, the estimated strength matrix $\left({\hat{W}}_{ji}\right)$ is updated according to the following law:

(51) $$\begin{array}{c} {\dot{\hat{W}}}_{ji}=-\Gamma_{i}\Omega_{j}\left(z\right){ℯ}^{T}P{\overset{ˇ}{B}}_{i}, \end{array}$$

where Γ_*i*_ denotes a positive definite matrix with the symmetric property.

## 6. Stability Analysis of the LQR-Based Neural-Fuzzy Control

In this section, the Lyapunov function is presented to analyze the global stability of the proposed control scheme under the effect of parametric uncertainties and external disturbances. Consider the Lyapunov candidate function as follows:

(52) $$\begin{array}{c} V=\frac{1}{2}{ℯ}^{T}Pℯ+\overset{p}{\underset{i=1}{\sum }}\left({\tilde{W}}_{ji}^{T}\;\Gamma_{i}^{-1}{\tilde{W}}_{ji}\right), \end{array}$$

with

(53) $$\begin{array}{c} \;{\tilde{W}}_{ji}={\hat{W}}_{ji}-{\bar{W}}_{ji}, \end{array}$$

where ${\tilde{W}}_{ji}$ denotes the estimation error between the estimated strength matrix and the ideal constant strength matrix.

Differentiating Equation (52) and employing Equations (49) and (37), one can obtain

(54) $$\begin{array}{c} \dot{V}=-{ℯ}^{T}\left(Q+K^{T}RK\right)ℯ+2{ℯ}^{T}P{\overset{ˇ}{B}}_{i}\times \left({\hat{d}}_{i}-{\overset{¯}{W}}_{ji}^{T}\;\Omega_{j}\left(z\right)-{\overset{¯}{\varrho }}_{i}\left(z\right)\right)+2\overset{p}{\underset{i=1}{\sum }}\left({\tilde{W}}_{ji}^{T}\;\Gamma_{i}^{-1}{\dot{\tilde{W}}}_{ji}\right). \end{array}$$

Now utilizing Equation (53), the error difference between the actual value and the desired value by the designed neural-fuzzy network can be expressed as

(55) $$\begin{array}{c} {\tilde{W}}_{ji}\Omega_{j}\left(z\right)={\hat{W}}_{ji}\Omega_{j}\left(z\right)-{\bar{W}}_{ji}\Omega_{j}\left(z\right). \end{array}$$

Moreover, as the firing strength matrix $\left({\bar{W}}_{ji}\right)$ is a constant matrix, Equation (53) holds the following relation after differentiation:

(56) $$\begin{array}{c} {\dot{\tilde{W}}}_{ji}={\dot{\hat{W}}}_{ji}. \end{array}$$

Reconstituting Equation (54) using Equations (55) and (56), one can obtain

(57) $$\begin{array}{c} \dot{V}=-{ℯ}^{T}\left(Q+K^{T}RK\right)ℯ+2{ℯ}^{T}P{\overset{ˇ}{B}}_{i}\times \left({\hat{d}}_{i}-{\hat{W}}_{ji}\Omega_{j}\left(z\right)+{\tilde{W}}_{ji}\Omega_{j}\left(z\right)-{\overset{¯}{\varrho }}_{i}\left(z\right)\right)+2\overset{p}{\underset{i=1}{\sum }}\left({\tilde{W}}_{ji}^{T}\;\Gamma_{i}^{-1}{\dot{\hat{W}}}_{ji}\right), \end{array}$$

(58) $$\begin{array}{c} \dot{V}=-{ℯ}^{T}\left(Q+K^{T}RK\right)ℯ+2\overset{p}{\underset{i=1}{\sum }}{ℯ}^{T}P{\overset{ˇ}{B}}_{i}\times \left({\hat{d}}_{i}-{\hat{W}}_{ji}\Omega_{j}\left(z\right)+{\tilde{W}}_{ji}\Omega_{j}\left(z\right)-{\overset{¯}{\varrho }}_{i}\left(z\right)\right)+2\overset{p}{\underset{i=1}{\sum }}\left({\tilde{W}}_{ji}^{T}\;\Gamma_{i}^{-1}{\dot{\hat{W}}}_{ji}\right). \end{array}$$

Now substituting Equations (50) and (51) into Equation (58), one can obtain

(59) $$\begin{array}{c} \dot{V}=-{ℯ}^{T}\left(Q+K^{T}RK\right)ℯ+2\overset{p}{\underset{i=1}{\sum }}{ℯ}^{T}P{\overset{ˇ}{B}}_{i}\times \left({\hat{d}}_{i}-{\hat{W}}_{ji}\Omega_{j}\left(z\right)-{\overset{¯}{\varrho }}_{i}\left(z\right)\right)\leq -{ℯ}^{T}\left(Q+K^{T}RK\right)ℯ\leq 0. \end{array}$$

Invoking the above equation, it can be concluded that the error dynamics of the coupled human-exoskeleton system is asymptotically stable. Therefore, the proposed controller carries out the asymptotic tracking with error **ℯ**⟶0 (as *t*⟶∞) following the disturbance estimator (Equation (50)) and firing strength adaptation law (Equation (51)). Furthermore, the local stability of the proposed controller can be analyzed using the pole placement theory, where the convergence rate can be investigated by keeping the poles on the left side of the *s*-plane [45].

## 7. Results and Discussion

In this section, the simulation results and analyses are presented to evaluate the effectiveness of the proposed control strategy (RLQR-NF) for an exoskeleton device during passive gait rehabilitation measures. The block representation for the proposed control strategy is schematically shown in Figure 7. At first, the performance of the proposed control strategy is compared with a contrast control strategy without parametric uncertainties and external disturbances. In this work, the exponential reaching law-based sliding mode (ERL-SM) control is used as a contrast control strategy [48]. Thereafter, two cases are contemplated to demonstrate the controller's robustness: the first case, increasing the coupled segment masses by 20% with a trigonometric form of disturbances, and the second case, increasing the coupled segment masses by 30% with a random form of disturbances.

### 7.1. Simulation Results without Parametric Uncertainties and External Disturbances

In this subsection, a comparative analysis between the RLQR-NF and ERL-SM control strategies is presented for desired gait tracking during passive gait rehabilitation measures. In the absence of parametric uncertainties and external disturbances, i.e., Δ = 0 and *d* = 0 in Equation (25), the nominal mass values of lower limb segments (*m*_t_ = 8.25, *m*_c_ = 3.85, and *m*_hf_ = 1.5) are taken into account for drawing the state of comparison. Using Equation (36), the optimal state gain matrix for the nominal mass parameters (*K*_8.25,3.85,1.5_) is calculated as below:

(60) $$\begin{array}{c} K_{8.25,3.85,1.5}=\left(\begin{array}{cccccc} 448.63 & -2.72 & -0.57 & 17.84 & -0.31 & -0.127\\ 7.65 & 12.40 & 2.49 & 3.20 & 20.27 & 0.82\\ 8.72 & -1.92 & 20.17 & 0.33 & -2.56 & 6.40 \end{array}\right). \end{array}$$

In the ERL-SM control strategy [48], the control law parameters are used as *c* = diag(50, 50, 50), *ε* = 0.5 × *I*_3_, and *k*_*e*_ = *I*_3_. As shown in Figure 8, the healthy gait trajectory is tracked by incorporating the kinematic and dynamic parameters into the proposed control (RLQR-NF) and ERL-SM control strategy. A time period of 2 seconds is considered to complete one gait cycle. The starting Cartesian position (*X*, *Y*: 0.25 m, -0.60 m) of the desired gait trajectory is illustrated in black color. The actual trajectories in the Cartesian coordinate frame are presented by the dashed blue line (RLQR-NF) and the green line (ERL-SM).

Figures 9(a) and 9(b) depict the tracking error in both directions, i.e., *X*- and *Y*-directions (**ℯ**_*x*_ and **ℯ**_*y*_). The maximum absolute deviation in the *X*-direction (|**ℯ**_*x*_|_max_) for the ERL-SM and RLQR-NF control schemes is 0.013 m and 0.008 m, respectively. In the *Y*-direction, the respective deviation (|**ℯ**_*y*_|_max_) is observed to be 0.009 m and 0.006 m for the ERL-SM and RLQR-NF control strategies.

The tracking of desired joint angles with applied control strategies is illustrated in Figures 10(a)–10(c). The angular deviations (**ℯ**_*θ*_H__, **ℯ**_*θ*_K__, and **ℯ**_*θ*_A__) from desired joint trajectories are shown in Figures 11(a)–11(c). Considering the hip joint, it is observed that the maximum absolute deviation (|**ℯ**_*θ*_H__|_max_) for respective controllers is 0.78° (ERL-SM) and 0.51° (RLQR-NF). In the knee joint, the deviation (|**ℯ**_*θ*_K__|_max_) is found to be 1.15° and 1.16° for the system with the ERL-SM and RLQR-NF control strategies, respectively. For the ankle joint, the respective deviations (|**ℯ**_*θ*_A__|_max_) are estimated as 0.81° (ERL-SM) and 0.32° (RLQR-NF).

Figures 12(a)–12(c) demonstrate the generated control signals (*u*_H_, *u*_K_, and *u*_A_) following the desired trajectory through repetitive gait rehabilitation exercises. With the ERL-SM control scheme, the peak values of the hip, knee, and ankle signals are estimated as 32.98 V, 19.88 V, and 1.8 V. On the other hand, with the RLQR-NF control scheme, the respective values of control signals are found to be 30.25 V, 18.1 V, and 1.25 V. It is evident from the results that the proposed control strategy (RLQR-NF) outperforms the contrast control strategy (ERL-SM) to track the desired gait trajectory, however, with a marginal difference. Therefore, to demonstrate the effectiveness of the proposed control when dealing with PUEDs, variations in mass parameters and the form of disturbances are considered further.

### 7.2. Simulation Results for Parametric Variations and External Disturbances

In order to realize the robustness of the proposed control strategy (RLQR-NF), the root mean square error (RMSE) is computed and compared with the ERL-SM control strategy for parametric uncertainties and external disturbances. Moreover, based on RMSE values, the performance index (PI) is calculated to analyze the improvement of the proposed control scheme over the contrast control scheme.

(61) $$\begin{array}{c} \text{RMSE}=\sqrt{\frac{1}{N}\overset{N}{\underset{a=1}{\sum }}{\left\|{ℯ}_{a}\right\|}^{2}},\\ \text{PI}=\frac{{\text{RMSE}}_{\text{ERL}‐\text{SM}}-{\text{RMSE}}_{\text{RLQR}‐\text{NF}}}{{\text{RMSE}}_{\text{ERL}‐\text{SM}}}\times 100\%, \end{array}$$

where **ℯ**_*a*_ : **ℯ**_*θ*_ represents the error between the desired and actual joint angles, and *N* is the size of the error vector. RMSE_ERL‐SM_ and RMSE_RLQR‐NF_ signify the root mean square errors related to ERL-SM and RLQR-NF control strategies.

Considering the first case of PUEDs (Case I), where the system masses are increased by 20% (*m*_t_ = 9.90, *m*_c_ = 4.62, and *m*_hf_ = 1.80) along with a trigonometric form of disturbances (*𝒟*_1_ = (6sin(4*πt*)), *𝒟*_2_ = (5sin(3*πt*)), and *𝒟*_3_ = (3sin(2*πt*))), the joint angular errors (**ℯ**_*θ*_H__, **ℯ**_*θ*_K__, and **ℯ**_*θ*_A__) for the applied control strategies are shown in Figures 13(a)–13(c). For the hip joint, RMSE_ERL‐SM_ and RMSE_RLQR‐NF_ are estimated as 0.578° and 0.283°, respectively. The respective RMSE values for the knee joint are found to be 0.672° and 0.42°. In ankle joint tracking, the RMSE values for the control strategies are recorded as 0.321° and 0.224°.

Considering the second case of PUEDs (Case II), where the system masses are increased by 30% (*m*_t_ = 10.73, *m*_c_ = 5.00, and *m*_hf_ = 1.95) along with a random form of disturbances (*D*_1_ = (5 × random(1)), *D*_2_ = (3 × random(1)), and *D*_3_ = (2 × random(1)), the joint angular errors (**ℯ**_*θ*_H__, **ℯ**_*θ*_K__, and **ℯ**_*θ*_A__) for the proposed and contrast control strategies are shown in Figures 14(a)–14(c). For the hip joint, the values of RMSE_ERL‐SM_ and RMSE_RLQR‐NF_ are found to be 0.613° and 0.287°, respectively. The respective RMSE values related to the knee joint tracking are obtained as 0.742° and 0.434°. The following RMSE values for the ankle joint are found to be 0.334° and 0.228°.

Table 5 presents the performance index (PI) of the proposed control over the contrast control. The proposed control is promising in desired gait tracking compared to the contrast control, subjected to PUEDs. Moreover, as observed from Table 5, the performance index (PI) is improved by 2.15%, 4.01%, and 1.52% in Case II as compared to Case I. During rehabilitation exercises, this performance investigation allows the lower limb exoskeleton system to carry out repetitive movements with greater accuracy under the presence of PUEDs.

The convergence of both control schemes is investigated by evaluating the settling time, i.e., the time lapsed for the error to drop within 2% of the final value. The settling time for the error in the hip, knee, and ankle joints for every set of mass values is presented in Table 6. The low values of settling time indicate the faster convergence of the proposed controller (RLQR-NF) over the contrast controller (ERL-SM) before achieving the full stable state.

## 8. Conclusions

In this work, a robust LQR-based neural-fuzzy control has been proposed to follow the natural gait trajectory using an exoskeleton system during passive rehabilitation measures. Primarily, a linearized state-space form of the nonlinear human-exoskeleton has been established via the input-output feedback linearization method. Employing the LQR state gain matrix, robust ANFIS training datasets have been formed with a variation of system parameters. The operating range of the error vector and control responses have been regarded as the training input and output vectors. The ANFIS architectures have been trained offline to deal with the effect of parametric uncertainties. Thereafter, the online adaptation law of firing strength in ANFIS architectures has been incorporated to deal with external disturbances. The asymptotic stability of the coupled dynamics while applying the proposed control has been ensured using the Lyapunov theory. Finally, the effectiveness of the proposed controller has been investigated by comparing it to the exponential reaching law-based sliding mode control. The robustness analysis has been carried out by varying mass parameters and inducing different forms of external disturbances. The simulation results have shown the potential of the proposed robust tracking control for passive gait rehabilitation using an exoskeleton system. In the future, the effect of human involvement will be considered to design an “assist-as-needed” control strategy during active rehabilitation.

## Figures and Tables

**Figure 1:** CAD model of (a) LLES (labels: (1) thigh link, (2) shank link, (3) foot link, (4) hybrid stepper motor, (5) lead screw actuator, (6) stepper motor, (7) timing belt, (8) support module, (9) wheels, and (10) telescopic link joint connector) and (b) LEES with a human dummy [32].

**Figure 2:** Gait analysis experiment. (a) Schematic diagram of the detailed procedure. (b) A child subject with the skeleton model during the experiment.

**Figure 3:** Experimental gait data. (a) Desired joint angular trajectory. (b) Desired gait trajectory.

**Figure 4:** Coupled human-exoskeleton configuration. (a) A simplified linkage model. (b) Interaction dynamics of the coupled human-exoskeleton system.

**Figure 5:** ANFIS architecture.

**Figure 6:** Flowchart representation of the stage-wise design procedure.

**Figure 7:** Schematic representation of the implemented proposed RLQR-NF controller.

**Figure 8:** Desired trajectory tracking for ERL-SM and RLQR-NF control schemes with nominal mass values.

**Figure 9:** Position tracking error for ERL-SM and RLQR-NF control schemes with nominal mass values. (a) *X*-direction. (b) *Y*-direction.

**Figure 10:** Joint angle tracking for ERL-SM and RLQR-NF control schemes with nominal mass values. (a) Hip joint. (b) Knee joint. (c) Ankle joint.

**Figure 11:** Joint tracking error for ERL-SM and RLQR-NF control schemes with nominal mass values. (a) Hip joint. (b) Knee joint. (c) Ankle joint.

**Figure 12:** Control signals for ERL-SM and RLQR-NF control schemes with nominal mass values. (a) Hip joint. (b) Knee joint. (c) Ankle joint.

**Figure 13:** Joint tracking error for ERL-SM and RLQR-NF control schemes with the first case of PUEDs. (a) Hip joint. (b) Knee joint. (c) Ankle joint.

**Figure 14:** Joint tracking error for ERL-SM and RLQR-NF control schemes with the second case of PUEDs. (a) Hip joint. (b) Knee joint. (c) Ankle joint.

**Table 1:** Specifications of the lower limb exoskeleton system and child dummy.

Part	Mass (kg)	Length (m)	COM (m)
Lower limb exoskeleton system			
Thigh link	*m*_1_^e^ = 4.75	*l*_1_^e^ = 0.25‐0.30	*l*_c1_^e^ = 0.12‐0.15
Shank link	*m*_2_^e^ = 1.60	*l*_2_^e^ = 0.30‐0.35	*l*_c2_^e^ = 0.14‐0.17
Foot link	*m*_3_^e^ = 0.85	*l*_3_^e^ = 0.05	*l*_c3_^e^ = 0.02

Child (age 8 years, body weight 30 kg, and body height 122 cm)			
Thigh	*m*_1_^h^ = 3.50	*l*_1_^h^ = 0.27	*l*_c1_^h^ = 0.13
Shank	*m*_2_^h^ = 2.25	*l*_2_^h^ = 0.30	*l*_c2_^h^ = 0.15
Foot	*m*_3_^h^ = 0.65	*l*_3_^h^ = 0.04	*l*_c3_^h^ = 0.02

**Table 2:** Variation in lower limb mass parameters of the coupled human-exoskeleton system.

Thigh, *m*_t_ (kg)	Calf, *m*_c_ (kg)	Heel-foot, *m*_hf_ (kg)
8.25	3.85	1.50
8.58	4.00	1.56
8.91	4.16	1.62
9.24	4.31	1.68
9.57	4.47	1.74
9.90	4.62	1.80

**Table 3:** Operating range of the error in state variables.

Variables in the error vector	Minimum value	Maximum value	Units
**ℯ**_*θ*_H__	-60	60	Degree
**ℯ**_*θ*_K__	-60	60	Degree
**ℯ**_*θ*_A__	-30	30	Degree
${ℯ}_{{\dot{\theta }}_{\text{H}}}$	-90	90	Degree/sec
${ℯ}_{{\dot{\theta }}_{\text{K}}}$	-90	90	Degree/sec
${ℯ}_{{\dot{\theta }}_{\text{A}}}$	-60	60	Degree/sec

**Table 4:** Training parameters of ANFIS architectures.

Training parameters	*anfis1*.*fis*	*anfis2*.*fis*	*anfis3*.*fis*
MF type	Gaussian	Gaussian	Gaussian
MF number	5	12	3
Error tolerance	0.00001	0.0001	0.001
Epochs	10	15	5
Learning model	Hybrid	Hybrid	Hybrid

**Table 5:** Comparative performance analysis of the proposed control over the contrast control.

Joint name	RMSE (ERL-SM) (deg)	RMSE (RLQR-NF) (deg)	PI (%)
Case I: with a 20% increment in mass parameters and a trigonometric form of external disturbances (*m*_t_ = 9.90, *m*_c_ = 4.62, and *m*_hf_ = 1.80)(*𝒟*_1_ = (6 × sin(4*πt*)), *𝒟*_2_ = (5 × sin(3*πt*)), and *𝒟*_3_ = (3 × sin(2*πt*)))			
Hip	0.578	0.283	51.04
Knee	0.672	0.420	37.50
Ankle	0.321	0.224	30.21

Case II: with a 30% increment in mass parameters and a random form of external disturbances (*m*_t_ = 10.73, *m*_c_ = 5.00, and *m*_hf_ = 1.95)(*𝒟*_1_ = (6 × random(4)), *𝒟*_2_ = (5 × random(3)), and *𝒟*_3_ = (3 × random(2))			
Hip	0.613	0.287	53.19
Knee	0.742	0.434	41.51
Ankle	0.334	0.228	31.73

**Table 6:** Settling time of ERL-SM and RLQR-NF control schemes for convergence analysis.

Control scheme	Lower limb joint	Settling time (sec)		
		Nominal system mass	Case I of PUEDs	Case II of PUEDs
ERL-SM	Hip	1.971	1.986	1.993
	Knee	1.962	1.974	1.988
	Ankle	1.927	1.943	1.969

RLQR-NF	Hip	1.951	1.967	1.991
	Knee	1.946	1.959	1.987
	Ankle	1.914	1.933	1.958

## Data Availability

The data used to support the findings of the study are included within the article.

## Appendix

The elements of the state-weight factor matrices (*A*, *B*) can be evaluated using the following derived formulations.

For the *A* matrix,

(A.1) $$\begin{array}{c} \alpha_{41}=-12l_{1}l_{2}l_{3}g\left(2m_{2}^{2}+4m_{1}m_{2}+3m_{1}m_{3}+2m_{2}m_{3}\right),\\ {\tilde{\alpha }}_{41}=2l_{2}l_{3}\left(12l_{1}^{2}m_{2}^{2}+12l_{1}^{2}m_{2}m_{3}+16l_{1}^{2}m_{1}m_{2}+12l_{1}^{2}m_{1}m_{3}-48l_{2}l_{3}m_{2}m_{3}-36l_{2}l_{3}m_{3}^{2}\right),\\ \alpha_{42}=72l_{1}l_{2}l_{3}g\left(m_{2}^{2}+m_{3}^{2}+2m_{2}m_{3}\right),\\ {\tilde{\alpha }}_{42}={\tilde{\alpha }}_{41},\\ \alpha_{43}=-18gl_{1}m_{2}m_{3},\\ {\tilde{\alpha }}_{43}=\frac{{\tilde{\alpha }}_{41}}{2l_{2}l_{3}},\\ \alpha_{51}=12g\left(6l_{1}m_{2}+3l_{1}m_{3}+4l_{2}m_{2}+3l_{2}m_{3}\right)\left(l_{1}m_{2}+l_{1}m_{3}+l_{2}m_{3}+\frac{l_{1}m_{1}}{2}+\frac{l_{2}m_{2}}{2}+\frac{l_{3}m_{3}}{2}\right),\\ {\tilde{\alpha }}_{51}={\tilde{\alpha }}_{51^{\prime \prime }}={\tilde{\alpha }}_{52^{\prime }}={\tilde{\alpha }}_{52^{\prime \prime }}={\tilde{\alpha }}_{53}={\tilde{\alpha }}_{53^{\prime \prime }}={\tilde{\alpha }}_{63}={\tilde{\alpha }}_{52}={\tilde{\alpha }}_{53^{\prime }}={\tilde{\alpha }}_{63^{\prime \prime }}=\frac{{\tilde{\alpha }}_{41}}{2l_{3}},\\ \alpha_{51^{\prime }}=6g\left(l_{2}m_{2}+2l_{2}m_{3}+l_{3}m_{3}\right)\left(4l_{1}^{2}m_{1}+12l_{1}^{2}m_{2}+3l_{1}^{2}m_{3}+4l_{2}^{2}m_{2}+3l_{2}^{2}m_{3}+12l_{1}l_{2}m_{2}+6l_{1}l_{2}m_{3}-12l_{2}l_{3}m_{3}\right),\\ {\tilde{\alpha }}_{51^{\prime }}=\frac{l_{2}{\tilde{\alpha }}_{41}}{2l_{3}},\\ \alpha_{51^{\prime \prime }}=6gm_{3}\left(6l_{1}^{2}l_{2}m_{1}+3l_{2}^{2}l_{1}m_{2}+9l_{1}^{2}l_{2}m_{2}+4l_{1}^{2}l_{3}m_{1}+12l_{1}^{2}l_{3}m_{2}+3l_{1}^{2}l_{3}m_{3}-12l_{3}^{2}l_{2}m_{3}-18l_{2}^{2}l_{3}m_{3}+6l_{1}l_{2}l_{3}m_{2}+3l_{1}l_{2}l_{3}m_{3}\right),\\ \alpha_{52}=6g\left(l_{2}m_{2}+2l_{2}m_{3}+l_{3}m_{3}\right)\left(6l_{1}m_{2}+3l_{1}m_{3}+4l_{2}m_{2}+3l_{2}m_{3}\right),\\ \alpha_{52^{\prime }}=6g\left(l_{2}m_{2}+2l_{2}m_{3}+l_{3}m_{3}\right)\left(4l_{1}^{2}m_{1}+12l_{1}^{2}m_{2}+3l_{1}^{2}m_{3}+4l_{2}^{2}m_{2}+3l_{2}^{2}m_{3}+12l_{1}l_{2}m_{2}+6l_{1}l_{2}m_{3}-12l_{2}l_{3}m_{3}\right),\\ \alpha_{52^{\prime \prime }}=\alpha_{51^{\prime \prime }}=\alpha_{53}=\alpha_{63},\\ \alpha_{53^{\prime }}=6gl_{3}m_{3}\left(6l_{1}m_{2}+3l_{1}m_{3}+4l_{2}m_{2}+3l_{2}m_{3}\right),\\ \alpha_{53^{\prime \prime }}=6gl_{3}m_{3}\left(4l_{1}^{2}m_{1}+12l_{1}^{2}m_{2}+3l_{1}^{2}m_{3}+4l_{2}^{2}m_{2}+3l_{2}^{2}m_{3}+12l_{1}l_{2}m_{2}+6l_{1}l_{2}m_{3}-12l_{2}l_{3}m_{3}\right),\\ \alpha_{61}=6g\left(l_{2}m_{2}+2l_{2}m_{3}+l_{3}m_{3}\right)\left(6l_{1}^{2}l_{2}m_{1}+3l_{2}^{2}l_{1}m_{2}+9l_{1}^{2}l_{2}m_{2}+4l_{1}^{2}l_{3}m_{1}+12l_{1}^{2}l_{3}m_{2}+3l_{1}^{2}l_{3}m_{3}-12l_{3}^{2}l_{2}m_{3}-18l_{2}^{2}l_{3}m_{3}+6l_{1}l_{2}l_{3}m_{2}+3l_{1}l_{2}l_{3}m_{3}\right),\\ {\tilde{\alpha }}_{61}={\tilde{\alpha }}_{61^{\prime }}={\tilde{\alpha }}_{62}={\tilde{\alpha }}_{62^{\prime }}={\tilde{\alpha }}_{63^{\prime }}=\frac{l_{2}{\tilde{\alpha }}_{41}}{2},\\ \alpha_{61^{\prime }}=6g\left(3l_{1}^{2}l_{2}^{2}m_{2}^{2}+12l_{1}^{2}l_{2}^{2}m_{2}m_{3}+4l_{1}^{2}l_{2}^{2}m_{1}m_{2}+12l_{1}^{2}l_{2}^{2}m_{1}m_{3}+18l_{1}^{2}l_{2}l_{3}m_{2}m_{3}+12l_{1}^{2}l_{2}l_{3}m_{1}m_{3}+12l_{1}^{2}l_{3}^{2}m_{2}m_{3}+3l_{1}^{2}l_{3}^{2}m_{3}^{2}+4l_{1}^{2}l_{3}^{2}m_{1}m_{3}-12l_{2}^{3}l_{3}m_{2}m_{3}-36l_{2}^{3}l_{3}m_{3}^{2}-36l_{2}^{2}l_{3}^{2}m_{3}^{2}-12l_{3}^{3}l_{2}m_{3}^{2}\right),\\ \alpha_{61^{\prime \prime }}=36gl_{1}\left(l_{2}m_{2}+2l_{3}m_{2}+l_{3}m_{3}\right)\left(l_{1}m_{2}+l_{1}m_{3}+l_{2}m_{3}+\frac{l_{1}m_{1}}{2}+\frac{l_{2}m_{2}}{2}+\frac{l_{3}m_{3}}{2}\right),\\ {\tilde{\alpha }}_{61^{\prime \prime }}={\tilde{\alpha }}_{62^{\prime \prime }}=\frac{{\tilde{\alpha }}_{41}}{2},\\ \alpha_{62}=\alpha_{61},\\ \alpha_{62^{\prime }}=\alpha_{61^{\prime }}=\alpha_{63^{\prime }},\\ \alpha_{62^{\prime \prime }}=36gl_{1}\left(l_{2}m_{2}+2l_{3}m_{2}+l_{3}m_{3}\right)\left(l_{2}m_{3}+\frac{l_{2}m_{2}}{2}+\frac{l_{3}m_{3}}{2}\right),\\ \alpha_{63^{\prime \prime }}=18gl_{1}m_{3}\left(l_{2}m_{2}+2l_{3}m_{2}+l_{3}m_{3}\right). \end{array}$$

For the *B* matrix,

(A.2) $$\begin{array}{c} \beta_{41}=96l_{2}l_{3}m_{2}+72l_{2}l_{3}m_{3},\\ {\tilde{\beta }}_{41}={\tilde{\alpha }}_{41},\\ \beta_{42}=-\left(144l_{1}l_{3}m_{2}+72l_{1}l_{3}m_{3}+96l_{2}l_{3}m_{2}+72l_{2}l_{3}m_{3}\right),\\ {\tilde{\beta }}_{42}={\tilde{\beta }}_{43}={\tilde{\beta }}_{41},\\ \beta_{43}=72l_{1}l_{2}m_{2}+144l_{1}l_{3}m_{2}+72l_{1}l_{3}m_{3},\\ \beta_{51}=-\left(72l_{1}m_{2}+36l_{1}m_{3}+48l_{2}m_{2}+36l_{2}m_{3}\right),\\ {\tilde{\beta }}_{51}=\frac{{\tilde{\beta }}_{41}}{2l_{3}},\\ \beta_{52}=48l_{1}^{2}m_{1}+144l_{1}^{2}m_{2}+36l_{1}^{2}m_{3}+48l_{2}^{2}m_{2}+36l_{2}^{2}m_{3}+144l_{1}l_{2}m_{2}+72l_{1}l_{2}m_{3}-144l_{2}l_{3}m_{3},\\ {\tilde{\beta }}_{52}=\frac{l_{2}{\tilde{\beta }}_{41}}{2l_{3}},\\ \beta_{53}=-\left(72l_{1}^{2}l_{2}m_{1}+36l_{2}^{2}l_{1}m_{2}+108l_{1}^{2}l_{2}m_{2}+48l_{1}^{2}l_{3}m_{1}+144l_{1}^{2}l_{3}m_{2}+36l_{1}^{2}l_{3}m_{3}-144l_{3}^{2}l_{2}m_{3}-216l_{2}^{2}l_{3}m_{3}+72l_{1}l_{2}l_{3}m_{2}+36l_{1}l_{2}l_{3}m_{3}\right),\\ {\tilde{\beta }}_{53}=\frac{l_{2}{\tilde{\beta }}_{41}}{2},\\ \beta_{61}=36l_{1}\left(l_{2}m_{2}+2l_{3}m_{2}+l_{3}m_{3}\right),\\ {\tilde{\beta }}_{61}=\frac{{\tilde{\beta }}_{41}}{2},\\ \beta_{62}=\beta_{53},\\ {\tilde{\beta }}_{62}={\tilde{\beta }}_{53},\\ \beta_{63}=36l_{1}^{2}l_{2}^{2}m_{2}^{2}+144l_{1}^{2}l_{2}^{2}m_{2}m_{3}+48l_{1}^{2}l_{2}^{2}m_{1}m_{2}+144l_{1}^{2}l_{2}^{2}m_{1}m_{3}+216l_{1}^{2}l_{2}l_{3}m_{2}m_{3}+144l_{1}^{2}l_{2}l_{3}m_{1}m_{3}+144l_{1}^{2}l_{3}^{2}m_{2}m_{3}+36l_{1}^{2}l_{3}^{2}m_{3}^{2}+48l_{1}^{2}l_{3}^{2}m_{1}m_{3}-144l_{2}^{3}l_{3}m_{2}m_{3}-432l_{2}^{3}l_{3}m_{3}^{2}-432l_{2}^{2}l_{3}^{2}m_{3}^{2}-144l_{3}^{3}l_{2}m_{3}^{2},\\ {\tilde{\beta }}_{63}=\frac{l_{2}l_{3}m_{3}{\tilde{\beta }}_{41}}{2}. \end{array}$$
